RETRACTED

# Physiochemical and Phytochemical Properties of Wax Apple (*Syzygium samarangense* [Blume] Merrill & L. M. Perry var. Jambu Madu) as Affected by Growth Regulator Application

**DOI:** 10.1100/2012/728613

**Published:** 2012-06-04

**Authors:** Mohammad Moneruzzaman Khandaker, Amru Nasrulhaq Boyce, Normaniza Osman, ABM Sharif Hossain

**Affiliations:** ^1^Institute of Biological Sciences, Faculty of Science, University of Malaya, 50603 Kuala Lumpur, Malaysia; ^2^Program of Biotechnolgy, Department of Biology, Faculty of Sciecne, University of Hail, Hail-2404, Saudi Arabia

## Abstract

This study represents the first paper of the effects of growth regulators on the physiochemical and phytochemical properties of the wax apple fruit, a widely cultivated fruit tree in southeast Asia. Net photosynthesis, sucrose phosphate synthase (SPS) activity, peel color, fruit firmness, juice content, pH value, total soluble solids (TSSs), and the sugar acid ratio were all significantly increased in growth regulators (PGRs) treated fruits. The application of gibberellin (GA_3_), naphthalene acetic acid (NAA), and 2,4-dichlorophenoxy acetic acid (2,4-D) significantly reduced titratable acidity and increased total sugar and carbohydrate content compared to the control. The 50 mg/L GA_3_, 10 mg/L NAA, and 5 mg/L 2,4-D treatments produced the greatest increases in phenol and flavonoid content; vitamin C content was also higher for these treatments. PGR treatment significantly affected chlorophyll, anthocyanin, and carotene content and produced higher phenylalanine ammonia lyase (PAL) and antioxidant activity levels. There was a positive correlation between peel color and TSS and antioxidant activity and both phenol and flavonoid content and PAL activity and anthocyanin formation. A taste panel assessment was also performed, and the highest scores were given to fruits that had been treated with GA_3_ or auxin. The study showed that application of 50 mg/L GA_3_, 10 mg/L NAA, and 5 mg/L 2,4-D once a week from bud development to fruit maturation increased the physiochemical and phytochemical properties of wax apple fruits.

## 1. Introduction

The wax apple, or *jambu air madu,* as it is known in Malaysia, is a nonclimacteric tropical fruit in the Myrtaceae family and is botanically identified as *Syzygium samarangense *[1]. Wax apple is widely cultivated throughout Malaysia, mainly in smallholdings ranging from 1 to 5 ha, with a total hectare estimated at 1,500 ha in 2005 [2]. It is also grown throughout the southeast Asian countries, such as Thailand, Indonesia, and Taiwan as well as other tropical countries. In Malaysia, there are three species which bear edible fruits, namely, the water apple *(Syzygium aqueum)*, Malay apple (*Syzygium malaccense*), and wax apple or *jambu air* (*Syzygium samarangense*). *S. samarangense* is the most popular of the three in southeast Asia, and the trees are cultivated in home gardens, often planted along driveways and paths. Fruit production is nonseasonal and the peak periods are in February to April and October to December. It has become an increasingly popular fruit in the tropical region where it can fetch a price of up to 3USD per kilogram and has the potential to bring great benefit to local farmers and the country's economy.

 The pear-shaped fruits are usually pink, light red, or red but may be greenish-white or cream-colored, and are generally crisp, often juicy, refreshing, with a subtly sweet taste and aromatic flavor. Wax apple fruits are eaten raw with salt or cooked as a sauce. Almost all of the fruit is edible. The fruit pulp is a rich source of phenolics, flavonoids and several antioxidant compounds and as a result is believed to have great potential benefits for human health. In addition to its use as food, it has also been used in traditional medicine for a variety of illnesses and conditions. The fruit can be used to treat high blood pressure and several inflammatory conditions, including sore throat, and can also be used as an antimicrobial, antiscorbutic, carminative, diuretic, and astringent. 

RETRACTED

It is important for fruit growers to have information on the differences in fruit quality among the available fruit varieties and the changes occurring in fruit quality parameters over time. PGRs enhance the rapid changes in physiological and biochemical characters and improve crop productivity. GA_3_ has been found to increase fruit firmness, color, yield, and soluble solid content [3]. NAA has been shown to significantly increase fruit yield, total soluble solids (TSSs), total sugar content, fruit color in Bing cherry, and vitamin C in guava fruits [4]. Synthetic auxin increases total antioxidant capacity and nutritional quality in transgenic Silcora seedless grape [5]. It was also reported that 2,4-D increased total sugar content and enhanced the activities of antioxidant enzymes [6]. The application of 2,4-D, GA_3_, and NAA significantly reduced acidity percentage and increased vitamin C content of citrus fruits [7]. It has been reported that GA_3_ significantly promotes the secondary metabolites, which affect the biosynthesis of flavonoids [8], hormonal regulation of anthocyanin formation, and enhancement of phenylalanine ammonia lyase (PAL) [9].

Currently, there is no available literature describing the effects of growth regulators on wax apple quality. This study investigated the effects of gibberellin and synthetic auxin on fruit quality and on the physiochemical and phytochemical properties of wax apple under field conditions. It is proposed that the application of PGRs can affect or promote the physiochemical and phytochemical quality of the wax apple fruit.

RETRACTED

## 2. Materials and Methods

### 2.1. Experimental Site

The experiments were performed in orchards located at Malaysian Agricultural Research and Development Institute (MARDI), Klang (2°30 N, 112°30 E), and at a commercial farm in Banting (1°28 N, 111°20 E), Malaysia, both at an elevation of approximately 45 m above sea level. The area under study has a hot and humid tropical climate. The soil in both orchards is peat, with a mean pH of approximately 4.6. The experiments were conducted between 2008 and 2011. The first season (December 2008–April 2009) of experiments was performed at MARDI, Jalan Kebun, Klang, and the second (May 2010–October 2010) and third (December 2010–May 2011) seasons' experiments were conducted at the farm in Banting. 

### 2.2. Treatment Application and Fruit Harvesting

Twelve-year-old wax apple plants were selected for the study. The trees were planted in a 4.2 m × 4.2 m hexagonal pattern and received the same horticultural management. Total-seventy of two trees were used for 1st season for GA_3_, NAA, and 2,4-D. Three hundred sixty uniform branches (five branches per tree), with approximately the same length, diameter, and number of leaves, were selected for sample branches for the GA_3_, NAA, and 2,4-D experiments. Similarly, same numbers of trees and uniform branches were selected for the second and third seasons. Different trees from two experimental sites were utilized for the different treatments in different years to avoid additive effects of growth regulators. Each experiment consisted of four treatments, including the control, in six replicates. The leaves, flowers, and young small fruits of selected uniform branches were sprayed with 20, 50, and 100 mg/L GA_3,_ 5, 10, and 20 mg/L NAA and 2,4-D and water (the control) once each week from the beginning of flower opening until fruit maturation. A total of seven spraying times were carried out; two times before anthesis and five times after anthesis, and 250 mL hormone solution was used per treatment (30 branches). It takes ten weeks from bud development to fruit ripening, and all the fruits were harvested eight weeks after anthesis. Immediately after harvest, all fruits were aggregated, sub-sampled and kept in a 4°C refrigerator until completion of the analysis.

### 2.3. Measurement of Physiological, Biochemical and Phytochemical Parameters

#### 2.3.1. Peel Color, Pulp Firmness, Juice and pH

The peel color of the fruits was measured using a Minolta colorimeter (CR-300, Konica, Japan). Parameters such as “*L*” (lightness), “*a*” (greenness to redness) and “*b*” (blueness to yellowness) were determined at three different spots around the top, middle and end of the fruits. Sample averages were calculated and the color was expressed in L*, a*, b* Hunter parameter, using the following formula (L* × a*)/b*. Fruit firmness was determined with a digital hand-held penetrometer (Model KM-1, Fujiwara, Japan). The fruit juice of each harvested fruit was extracted and weighed, and the average juice weight was calculated separately for each treatment. The pH of the wax apple juice was recorded using a pH meter (Hanna pH 211, Italy). 

RETRACTED

#### 2.3.2. Titratable Acidity and Sugar Acid Ratio

The fruit juice (10 mL) was titrated with 0.1 M NaOH, and the results are expressed in terms of percentage citric acid. The percentage of citric acid was calculated using the formula of Bhattarai and Gautam [10], and the sugar acid ratio of the wax apple juice is given as the ratio of TSS/TA:

(1) $$\text{TA}\left(\%\right)=\frac{N_{b}\times V_{b}\times E_{a}\times \text{df}\times 100}{V_{s}},$$

where *N*_*b*_ is normality of the base, *V*_*b*_ is volume of the base, *E*_*a*_ is mill equivalent weight of citric acid, *V*_*s*_ is volume of sample, and df: dilution factor. 

#### 2.3.3. Determination of Soluble Carbohydrates and Total Sugar

The total soluble solids (TSSs) value was determined at 25°C with an Atago 8469 hand refractometer (Atago Co. LTD., Tokyo, Japan) and expressed as °Brix. Glucose, fructose, and sucrose were evaluated at 25°C with the HI 96811 digital refractometer (Hanna instruments) and expressed as percentages. Total soluble sugar was determined using the phenol-sulfuric method [11].

#### 2.3.4. Determination of Vit-C, Polyphenolic Compounds, and Pigment Concentration

Total ascorbic acid (vit-C) content was determined using the method modified by Hashimoto and Yamafuji [12]. The total phenolic contents (TPC) of wax apple fruits were determined with the Folin-Ciocalteu assay, as described by Singleton and Rossi [13]. Total flavonoid content (TFC) was determined with the aluminum chloride colorimetric assay, using catechin as a standard [14]. The chlorophyll and carotene contents of the leaves and fruit were determined using the methods described by Hendry and Price [15]. The total anthocyanin and carotenoid contents of the hydrophilic extracts were measured using the pH-differential method with cyanidin-3-glucoside used as a standard, as described by Rodríguez-Saona et al. [16]. 

#### 2.3.5. 2,2-Diphenyl-1-picryhydrazyl (DPPH) and 2,2′-azinobis-3-ethylbenzothiazoline-6-sulfonic Acid (ABTS) Free-Radical-Scavenging Assays

The DPPH free-radical scavenging activity was determined as described in Yang et al. [17]. The ABTS free-radical-scavenging activity was determined as described in Re et al. [18].

RETRACTED

#### 2.3.6. PAL Enzyme Activity and Taste Panel Evaluation

PAL activity in the crude enzyme extracts was assayed using the method described by Zucker [19] and expressed as nmol cinnamic acid yield. To evaluate the overall sensory characteristics of the wax apple fruits from various treatments, a taste panel was performed with twelve panelists. All panelists had been previously trained with the specific sensory evaluation test. They evaluated the randomly offered fruits on a scale from 0 to 100 (low-high scores for each evaluated variable) based on the following criteria: taste, flavor, color, firmness, acidity, sweetness, mouth aroma, and taste remaining after swallowing.

**Net Photosynthesis, Enzyme Extraction, and SPS Assay**

Treated wax apple leaf samples (0.5 g) were homogenized in 2 mL of ice-cold 50 mM MOPS-KOH buffer (pH 7.3), 5 mM MgCl_2_, 1 mM ethylene diamine tetra acetic acid (EDTA), 16 mM mercaptoethanol, 0.1% (v/v) Triton X-100, 10% (v/v) glycerol, 2 mM benzamidine, 1 mgL^−1^ leupeptin, and 2 mM phenylmethyl-sulfonyl fluoride. The crude extract (0.8 mL) was desalted by centrifugal gel filtration using a 4 mL Sephadex-G25 (Pharmacia) column equilibrated with 50 mM MOPS-KOH (pH 7.3), 5 mM MgCl_2_, 1 mM EDTA, 16 mM mercaptoethanol, and 10% (v/v) glycerol. The desalted crude extract was used for enzyme analysis, and protein content was determined by Bradford method [20] using bovine serum albumin as standard. SPS activity was assayed under *V*_max⁡_ condition as described by Huber et al. [21]. The photosynthesis rate (*Pn*) was measured using an Li-6400XT portable photosynthesis system (Li-COR Biosciences, Lincoln, NE, USA). Measurements were made immediately after treatment application at 9.00 am to 1.00 pm, and fifty four leaves were selected from GA_3_ and NAA treatments and control branches. Before measuring the photosynthetic parameter, the cuvette chamber conditions were set to provide photosynthetic photon flux density of 400, 800, 1200, and 2000 *μ*mol m^−2^ s^−1^ and cuvette block temperature was maintained at 24°C, and the concentration of CO_2_ was set at 350 *μ*mol mol^−1^ with a flow rate of 500 mL s^−1^.

### 2.4. Statistical Analysis

The experimental design was a randomized complete block design (RCBD) with six replications. The data obtained from three successive seasons were pooled and analysed using MSTAT-C statistical software. A one-way ANOVA was applied to evaluate significant differences in the studied parameters in the different treatments. The least significant difference (Fisher's protected LSD) was calculated following a significance *F*-test (at *P* = 0.05).

RETRACTED

## 3. Results

### 3.1. Peel Color Development

Fruit color is considered to be one of the important external factors in determining fruit quality, as the appearance of fruit greatly influences consumer's preferences.  Table 1 shows that fruit color development was greatly enhanced by the PGRs treatments. In the “4th” week of observation, fruits treated with 50 mg/L GA_3_ showed a*, b* value 99, followed by fruits treated with 100 and 20 mg/L GA_3_, whereas control fruits had only a*, b* value 30. The difference between the treatments and control was statistically significant (Table 1). For NAA treatments, fruits treated with 10 mg/L showed a*, b* value 80. In contrast, control fruits had only a*, b* value 30, and the differences between the treatments and the control were statistically significant. The application of 2,4-D also had a significant effect on peel color development of wax apple fruits (Table 1).

### 3.2. Pulp Firmness, Juice Content, and pH of Fruit Juice

The pulp firmness of wax apple fruits treated with different growth regulators is presented in Table 1. The pulp firmness of wax apple fruits was significantly affected by PGR application. Our results showed that pulp firmness increased with growth regulator application. The highest pulp firmness was recorded in fruits treated with 10 mg/L NAA, 50 mg/L GA_3_, and 10 mg/L 2,4-D,with measured values of 8.0, 7.5, and 7 (N), respectively. The pulp firmness of untreated fruit was 6.5 (N). The results show that the highest amount of juice (81 mL/100 g) was obtained in 50 mg/L GA_3_-treated fruits. The next-highest quantities were obtained in fruits treated with 20 and 100 mg/L, with juice percentages of 80 and 78 mL/100 g, respectively. The lowest juice percentage of 69 mL/100 g was obtained in the control. The differences between the treatments and control were statistically significant. Synthetic auxin (NAA or 2,4-D) treatments also produced significant effects on juice content in wax apple fruits. As shown in Table 1, the pH of the fruit juice was affected by growth regulator application, and the pH values of the juice fell within the range of 4.9–5.29. The differences in pH were statistically significant between the GA_3_ treatments and control. The results show that the highest pH (5.29) was recorded for the 50 mg/L GA_3_ treatment, while the lowest pH value (4.9) was recorded in the control. For the NAA, and 2,4-D treatments, the highest pH values (5.15 and 5.12) were recorded for the 10 mg/L 2,4-D and NAA treatments, respectively. The control pH value was the lowest (4.9), and the differences in pH value were statistically significant between the treatments and control.

RETRACTED

### 3.3. Titratable Acidity (TA) and Sugar Acid Ratio

The results for the TA experiments are shown in Table 1. Our results clearly indicate that titratable acidity was significantly affected by growth regulator application. The lowest amount of TA (0.70%) was observed with the 100 mg/L GA_3_ treatment, followed by the TA amounts for the 50 and 20 mg/L GA_3_ treatments. The highest amount of titratable acidity (0.78%) was observed in the control. Similarly, significant changes in titratable acidity of wax apple fruits were recorded with NAA and 2,4-D application, and the lowest amount (0.71%) was recorded with the 20 mg/L NAA treatment. As shown in Table 1, the sweetness index (sugar acid ratio) of fruits was significantly enhanced by the GA_3_, NAA and 2,4-D treatments. The 50 mg/L GA_3_ treatment increased the sugar acid ratio by 87%, followed by the 10 mg/L NAA and 10 mg/L 2,4-D treatments with increases of 71% and 60%, respectively, relative to the control.

### 3.4. TSS, Soluble Carbohydrates, and Total Sugar

TSS is an important quality factor attribute for many fresh fruits during ripening. The solids include acids and the soluble sugars sucrose, glucose, and fructose. As shown in Table 2, the highest TSS value of 11.5 (°Brix) was observed in 50 mg/L GA_3_-treated fruit, followed by fruit treated with 100 and 20 mg/L GA_3_ treatments, with TSS values of 10.1 and 9.07, respectively. The minimum TSS in the control samples was 6.70 (°Brix). NAA and 2,4-D treatments also produced higher TSS contents than the control, and the differences were statistically significant (Table 2). Carbohydrates, namely glucose, fructose, and inverted sugar, were evaluated in this study. The carbohydrate content of wax apple fruits was significantly elevated by GA_3_ and NAA application. The highest glucose, fructose and inverted sugar contents were observed in the fruits treated with 50 mg/L and 5 mg/L NAA. The control samples contained the lowest amounts of glucose, fructose, and inverted sugar. Nonsignificant changes in carbohydrate content were observed with the 2,4-D treatments (Table 2). After performing the above experiments, we determined the sugar contents of the wax apple fruits. For the GA_3_ treatments, statistically significant differences between the treatments and control were observed. The results for GA_3_ are shown in Table 2, and the highest total sugar content of 6.5 g/100 g was recorded for the 50 mg/L GA_3_-treated fruits, followed by the 100 and 20 mg/L GA_3_-treated fruits, with sugar contents of 5.82 and 5.57 g/100 g, respectively. In contrast, the control fruits showed the lowest sugar content of 3.65 g/100 g. Significant changes in total sugar content were also observed with NAA and 2,4-D application (Table 2).

RETRACTED

### 3.5. Vit-C Content

In this study, growth regulator application significantly affected the vit-C content of wax apple fruits (Table 3). With GA_3_ application, the highest vit-C content (6.6 mg/100 g) was recorded in 50 mg/L treated fruits, followed by fruits treated with 20 and 100 mg/L GA_3_, with vit-C contents of 5.9 and 5.8 mg/100 g, respectively. The lowest amount of vit-C (5.1 mg/100 g) was recorded in control fruit. Similarly, significant increases in vit-C content were observed in wax apple fruits treated with NAA and 2,4-D. The highest vit-C contents for auxin application were observed in the 5 mg/L NAA and 2,4-D treatments, with 6 and 5.6 mg/100 g, respectively.

### 3.6. Total Phenol and Flavonoid Content

As shown in Table 3 the TPC and TFC contents were clearly increased following growth regulator application. For GA_3_ treatment, the highest phenol and flavonoid contents (535 mg GAE/100 g and 45 mg CE/100 g, resp.) were recorded with the 50 mg/L GA_3_ treatment, followed by contents recorded in the 20 and 100 mg/L treatments. The control had the lowest levels of phenols and flavonoids (311 mg GAE/100 g and 18.5 mg CE/100 g, resp.). The differences between the treatments and control were statistically significant. Significant changes in the phenol and flavonoid contents of wax apple fruits were also observed with NAA and 2,4-D treatments. The effect of 2,4-D treatment on phenol and flavonoid content was highest with lower concentrations of 2,4-D (Table 3). Higher concentrations of 2,4-D showed a negative effect on the phytonutrient content of wax apple fruits.

### 3.7. Degradation of Chlorophyll

Chlorophyll content of ripening wax apple skin was also observed in this study. The results show that GA_3_, NAA, and 2,4-D application significantly reduced the chlorophyll content in fruits. The highest chlorophyll content (0.63 mg/L) was observed in the control, followed by amounts recorded in the 20 and 100 mg/L GA_3_ treatments. The lowest amount (0.24 mg/L) was recorded in 50 mg/L GA_3_-treated fruits (Table 3). These results indicate that growth regulator application stimulates the pigmentation of wax apple fruits under field conditions. For NAA and 2,4-D application, nonsignificant changes in chlorophyll content were observed.

### 3.8. Anthocyanin and Carotenoid Biosynthesis

As shown in Table 3, the application of various growth regulators had significant effects on the anthocyanin and carotene contents in wax apple fruits. For GA_3_ treatment, the highest amount of anthocyanin (46.0 mg/100 g) was observed with the 50 mg/L GA_3_ treatment, followed by the 20 and 100 mg/L treatments, with values of 40.0 and 36.0 mg, respectively. The control fruits had the lowest anthocyanin content (24.3 mg/100 g). NAA and 2,4-D treatments also produced significant changes in anthocyanin content (Table 3). The results show that the 50 mg/L GA_3_ treatment nearly doubled the carotenoid content in wax apple fruits. For NAA treatment, the highest carotenoid content (10.5 *μ*g/g) was observed with the 10 mg/L NAA treatment, followed by the 5 and 20 mg/L NAA treatments, with carotene contents of 9.83 and 8.90 *μ*g/g, respectively. The carotenoid content was 5.97 *μ*g/g in control fruits (Table 3). Similar to the GA_3_ and NAA treatments, 2,4-D treatments also yielded higher carotenoids in the fruits.

RETRACTED

### 3.9. Antioxidant Content

The DPPH and ABTS radical scavenging activity measured in wax apple fruit extracts was affected by different growth regulators, as shown in Figure 1. Our results showed that the IC_50_ of the DPPH and ABTS radical scavenging activity increased with PGR application. The results showed that the DPPH and ABTS radical scavenging activity increased up to 70% and 54% in fruit extracts from the 50 mg/L GA_3_ treatment, while activity in the control was only 50% (Figures 1(a) and 1(a1)). For NAA treatments (Figures 1(b) and 1(b1)), the highest antioxidant capacity, determined using both the DPPH and ABTS assays, was observed in 10 mg/L NAA-treated fruits, followed by the 5 and 20 mg/L NAA-treated fruits. Control fruits showed the least antioxidant capacity. As with the 2,4-D treatments, 24% and 30% more DPPH and ABTS radical scavenging activity was recorded for extracts of 5 mg/L 2,4-D-treated fruits (Figures 1(c) and 1(c1)). Overall, GA_3_, NAA, and 2,4-D application increased the antioxidant capacity of wax apple fruits (Figure 1).

### 3.10. PAL Enzyme Activity of Fruits

Our results show that GA_3_ treatment had a significant effect on PAL activity of the treated fruits (Figure 2(a)). PAL activity, as measured by cinnamic acid yield, was highest (15.67 nmol-cinnamic acid min^−1^ mg protein^−1^) for the 50 mg/L GA_3_ treatment, followed by the 100 and 20 mg/L GA_3_ treatments, with PAL activity values of 10.59 and 9.39 nmol-cinnamic acid min^-1 ^mg protein^−1^, respectively. The lowest PAL activity (8.15 nmol-cinnamic acid min^−1^ mg protein^−1^) was recorded in the control. The synthetic auxins NAA and 2,4-D also produced significant differences in PAL activity (Figures 2(b) and 2(c)). For NAA, the highest PAL activity was recorded in 10 mg/L NAA-treated fruits, followed by fruits treated with 20 and 5 mg/L NAA. Control fruits produced the lowest amount of cinnamic acid (Figure 2(b)). Significant changes were similarly observed in 2,4-D-treated fruits (Figure 2(c)).

RETRACTED

### 3.11. Correlations between Peel Color and TSS and between Phenols and Antioxidant Activity, PAL Activity, and Anthocyanin Formation

Figure 3 shows the relationship between peel color and TSS and between phenol content and antioxidant capacity, determined using the DPPH and ABTS assays, in the wax apple fruits analyzed. A high degree of correlation (*R* ^2^ = 0.97 for 50 mg/L GA_3_, *R* ^2^ = 0.95 for 10 mg/L NAA, and *R* ^2^ = 0.93 for 5 mg/L 2,4-D) was observed for the peel color and TSS content of treated fruits. Similarly, a high degree of correlation (*R* ^2^ = 0.86 for 50 mg/GA_3_, *R* ^2^ = 0.92 for 10 mg/L NAA, and *R* ^2^ = 0.74 for 5 mg/L 2,4-D was observed for total phenols and antioxidant capacity (Figure 3). We also got positive correlation between PAL activity and anthocyanin formation in PGR-treated fruits (Figures 2(d), 2(e), and 2(f)).

### 3.12. Taste Panel Results on Overall Fruit Quality Attributes

A spider chart was constructed to diagram the overall fruit quality evaluation of the panelists and shows the evaluation grades for the various attributes tested in the panel (Figure 4). The results show that fruits from the 50 mg/L GA_3_ treatment were designated as having the best taste, mouth aroma, and highest sweetness and were also classified among those having the lowest acidity, best flavor, and best aftertaste. On the other hand, fruit from the 10 mg/L NAA and 5 mg/L 2,4-D treatments exhibited intermediate values for most of the attributes tested. The control fruits had the highest acidity and exhibited low values for aftertaste, appearance, and sweetness.

### 3.13. Net Photosynthesis and SPS Activity

To measure the activity level of photosynthetic carbon metabolism, we determined the photosynthetic activity in terms of *μ*mol CO_2_ fixed m^−2^ s^−1^. GA_3_ and NAA treatments increased the leaf photosynthesis activity considerably; this effect was statistically significant in the observations of the 2010-2011 season. The activities were 1.64-, 2.42-, and 2.57-fold higher than the control at 350 ppm CO_2_ and light intensities of 400, 800, and 2,000 *μ*mol m^−2^ s^−1^, respectively, in the leaves treated with 50 mg/L GA_3_ (Figure 2(a)). Leaf photosynthesis was highest with the 50 mg/L treatment, followed by the 100 and 20 mg/L GA_3_ treatments, in that order, whereas the control leaves evidenced the least photosynthesis. For NAA treatments, 10 mg/L treated plant showed highest photosynthetic activity compared to others and control. Sucrose phosphate synthase activity of treated leaves also increased significantly for GA_3_ and NAA treatments (Figures 2(b) and 2(d))

RETRACTED

## 4. Discussion

The colors, or pigments, in fruits and vegetables reflect the presence of certain biologically active phytochemical compounds and antioxidants that have been reported to promote good health. Positive values of a* and b*, as observed in this work, are attributed to carotenoids or anthocyanins present in the skin. Our results for peel color development are in agreement with those of Basak et al. [3] that application of GA_3_ increases the color of fruits. Raphael et al. [22] also observed that synthetic auxin enhanced fruit color development in Bing cherry fruit. The increase observed, as a result of growth regulator applications, is possibly due to an increase in the activity of enzymes responsible for color development. In our study, growth regulators had positive effects on the firmness of wax apple fruits. These findings are in agreement with those of Choi et al. [23] that GA_3_ increased fruit firmness at harvest and decreased the rate of fruit softening. Similar findings were reported by Iqbal et al. [4], who showed that application of synthetic auxin significantly increased pulp firmness in loquat fruit.

The amount fruit juice produced is normally related to fruit size and genetic characteristics of a particular fruit. It has also been documented in previous studies that growth regulators can have a significant effect on fruit size and as a consequence the amount of fruit juice. In this study GA_3_ treatment was found to have a positive effect on the juice content of wax apple fruits. These results are in agreement with those of Wang et al. [24] that the application of gibberellic acid at flowering and preharvest significantly increased the juice percentage in various citrus species. Synthetic auxin increases absolute juice content in citrus fruits, through simultaneous increases in fruit size and juice content from pulp [7]. We obtained similar results with NAA and 2,4-D in wax apple fruits. Data for fruit juice pH were in agreement with the findings of Thakur et al. [25] that the acidity of tomato fruits was reduced when the plant was sprayed with GA_3_ and 2,4-D. Thakur et al. [25] also reported, however, that ascorbic acid content increased with higher concentrations of 2,4-D. In the present study, growth regulator application significantly reduced the titratable acidity content in wax apple fruits. The reduction in titratable acidity observed, with the application of PGRs, can probably be attributed to the conversion of the organic acids to sugar during fruit ripening. Thakur et al. [25] similarly reported that titratable acidity was significantly reduced with GA_3_ and auxin application. GA_3_ application had a greater effect on reducing acidity compared to NAA. Our results for acidity percentage were in agreement with those of Xiao et al. [7] that application of PGRs significantly reduced acidity percentage. It is also important to note that acidity increased with increasing concentrations of 2,4-D (Table 1), indicating that 2,4-D should be applied at low concentrations for quality improvement.

RETRACTED

Wahdan et al. [26] reported that GA_3_ treatments significantly increased the TSS, sugar acid ratio, and total sugar content of mango, whereby the ratio of sugar and acid determines the taste, flavor, and acceptability of fruit. We also observed significant changes in the sugar acid ratio due to growth regulator application in wax apple fruits. In fact, the sugar acid ratio may be also the key factor affecting the quality of wax apple under tropical climates. In our study, GA_3_ and auxin treatments significantly increased the TSS (°Brix) content of wax apple. These results are in agreement with those of Basak et al. [3] that auxin and gibberellins significantly increased the TSS contents of the citrus fruits tested.

Carbohydrates, such as glucose, fructose, and sucrose, play a central role in metabolism and regulate many developmental and physiological processes in plants. We observed that gibberellin and auxin treatments significantly altered carbohydrate concentration in wax apple fruits. The results are in agreement with Wang et al. [24], who reported that application of 2,4-D, GA_3_, and some other growth regulators increased the sugar content in various mandarin and sweet orange cultivars. Synthetic auxin application during anthesis was found to increase the amount of sugar content in tomato [4]. Accordingly, in this study, also PGRs treatments produced significant effects on total sugar content of wax apple. PGRs treatments may influence the source-sink balance in a plant and as a result increase the accumulation rate of carbohydrate content in wax apple fruit.

Vit-C content in fruits varies among crop species and is affected by environmental factors, time of fruit harvesting, plant vigor, the age of the plant, and the use of growth regulators. In this study, we observed that GA_3_ treatments had a significant effect on vit-C content in wax apple. With respect to vit-C content, GA_3_ treatments were more beneficial compared to 2,4-D and NAA treatments, as vit-C content decreased with increasing concentrations of synthetic auxin (2,4-D or NAA). Our results were consistent with those of Xiao et al. [7] that preharvest application of growth regulators increased vit-C content of the citrus fruits.

RETRACTED

From our findings, GA_3_ treatments clearly had a significant effect on the total flavonoid and phenolic content of wax apple fruits. Our results also showed that phenolic content positively correlated with antioxidant activity in GA_3_-treated fruits. These results are in agreement with the findings of Pourmorad et al. [27] that the extracts of *M. officinalis* containing the highest amounts of flavonoid and phenolic compounds exhibited the greatest antioxidant activity. In our study, synthetic auxin also had a significant effect on the total phenolic content of wax apple fruits. This finding correlates with that of Elisa et al. [5] in that auxins increased the total polyphenolic content, as well as the nutritional content in grape. Flavonoids are ubiquitous plant secondary metabolites and play a vital role in their physiology by producing the red and purple anthocyanin pigments. The present study indicates that the flavonoid content of wax apple is significantly affected by PGRs and is consistent with the findings of Klessig and Malamy [8] that GA_3_ promote synthesis of flavonoids, as increased anthocyanin synthesis, promoted by GA_3_, was found to promote levels of flavonoid-specific mRNAs. Elisa et al. [5] also reported that the flavonoid content of grape was significantly affected by auxin application. It is believed that the applied growth regulators elevated the level and activity of chalcone synthase, an enzyme responsible for the synthesis of pigments and thus stimulated flavonoid synthesis in treated fruits.

In this study, it was observed that chlorophyll loss gradually occurred with PGRs application. Perez et al. [28] reported similar findings that the plant growth regulator methyl jasmonate promoted chlorophyll degradation in the skin of Golden Delicious apples. Our results indicate that growth regulators had positive effects on anthocyanin and carotenoids content in wax apple fruits. These results are in agreement with the findings of Roussos et al. [29] that anthocyanin content in strawberry fruit increased significantly when the plants were treated with GA_3_. These observations suggest that GA_3_ could also play a role in the accumulation of pigments in fruits. Our results for anthocyanin content with auxin treatment were in agreement with the findings of Teresa et al. [9] that growth regulators enhanced the accumulation of anthocyanin content in strawberry fruits.

Our results showed that fruit treated with PGRs exhibited higher antioxidant capacity than control fruits. These findings are consistent with the results of Klessig and Malamy [8] that GA_3_ and auxin significantly promoted biosynthesis of secondary metabolites in fruit with the highest antioxidant activity. PAL is one of the key enzymes controlling anthocyanin biosynthesis from phenylalanine. In our study, growth regulators had significant effects on PAL activity in wax apple fruits. This increased PAL activity probably contributed to the enhanced red color development observed in the growth regulator treated fruits. These results were consistent with those of Teresa et al. [9] that GA_3_ and auxin increased PAL activity in strawberry plants.

RETRACTED

Our results for peel color and TSS of treated fruits were in agreement with the results of Moneruzzaman et al. [30] that fruit color positively correlated with soluble solids in tomato. In this study, a positive correlation was observed between antioxidant activity and total phenolic and flavonoid content also PAL activity with anthocyanin synthesis. This correlation indicates that phenolic and flavonoid compounds could be the primary factors governing antioxidant activity in the wax apple fruit samples, in agreement with previous findings that many phenolic compounds in plants are good sources of natural antioxidants [31].

Many researchers have identified positive relationships between biochemical analysis data and taste panel results, including a correlation between the sweetness of fruits and their TSS [32]. The panelists graded 50 mg/L GA_3_-treated fruits as the sweetest, followed by the 10 mg/L and 5 mg/L 2,4-D-treated fruits. These results were in agreement with the highest TSS and sweetness index values having been observed in these treatments. Furthermore, the panelists classified fruits from these treatments as having the lowest acidity, greatest color, and best taste, again in agreement with the high sweetness index found for these fruits.

As is well known, during and after photosynthesis, sugars, namely sucrose, are exported from the source leaves to other plant parts. Sucrose is synthesised in the cytosol from triose phosphates made in the Calvin cycle and exported from the chloroplasts, where it is converted into fructose 6-phospate which combines with UDP glucose to form sucrose phosphate, catalysed by sucrose phosphate synthase. It has been shown in our study that GA_3_ and NAA treatments increased the net photosynthesis and SPS activity of wax apple plants (Figure 5). Hubbard et al. [33] also found positive relationships between SPS activity and sucrose accumulation in melon. PGRs treatments may also increase the invertage activity, the increase invertage activity suggests for sucrose synthesis and vice versa due to increased photosynthetic product in treated leaves. The increased SPS activity could raise not only sucrose level but also glucose and fructose level in leaves and fruits of wax apple. It is suggested from this study that PGRs treated fruits accumulated the high percentage of sugar, polyphenolic compound, and antioxidant substances in fruits, thus increase its taste, flavour, as well as quality.

RETRACTED

## 5. Conclusions

From the present study, we concluded that the PGRs (GA_3_, NAA, and 2,4-D) can improve the physiochemical and phytochemical status of wax apple fruits. Nevertheless, it must be emphasized that the positive effects of PGRs on the quality of wax apple are dependent on types, dose, and environmental conditions. 50 mg/L GA_3_ treatment produced greater increases in physiochemical and phytochemical nutrition than the 100 and 20 mg/L GA_3_ treatments. For NAA, the 10 mg/L NAA treatment had the greatest effect on physiochemical and phytochemical nutrition. For 2,4-D, another synthetic auxin, the most promising results were obtained with a low concentration of 5 mg/L, and treatments in excess of 10 mg/L actually produced adverse effects on physiochemical and phytochemical properties. Our results also showed that the treated fruits with the highest antioxidant content were also ranked most favorably for fruit quality attributes and taste. From experiments performed under field conditions, we concluded that the 50 mg/L GA_3_, 10 mg/L NAA, and 5 mg/L 2,4-D treatments show particular promise for enhancing the physiochemical and phytochemical quality of wax apple fruits.

## Figures and Tables

**Figure 1:** Changes in antioxidant activity: (a) and (a1) GA_3_ treated, (b) and (b1) NAA treated, (c) and (c1) 2,4-D treated wax apple fruits using the DPPH and ABTS assays. Vertical bars represent the LSD at the 5% level.

**Figure 2:** Effects of treatments of GA_3_ (a) and (d), NAA (b) and (e) and 2,4-D (c) and (f) on PAL activity and correlation between PAL and anthocyanin synthesis in wax apple fruits. Data are means of six replicates ± SE. Different letters represent the significance at the 5% level of LSD test.

**Figure 3:** Correlation between peel colour and TSS and total phenols and antioxidant capacity in the GA_3_, NAA, and 2,4-D treated fruits.

**Figure 4:** Taste panel scoring of fruits from the GA_3_, NAA and 2,4-D treatments, based on the examined quality attributes.

**Figure 5:** Effect of GA_3_ treatment on (a) SPS activity, (b) net photosynthesis and NAA treatment on (c) SPS activity, and (d) net photosynthesis of wax apple leaves. Data are means of six replicates ± SE. Different letters represent the significance at the 5% level of LSD test.

RETRACTED

**Table 1:** Effect of GA_3_, NAA and 2,4-D treatments on physicochemical properties of wax apple fruits.

Treatment (mg/L)	Peel color L*a*/b*	Pulp firmness (N)	Fruit juice (mL/100 g)	PH	TSS (°Brix)	Titratable acidity (%)
Control	30 ± 3.2^*b*^	6.5 ± 0.45^*b*^	69 ± 0.66^*b*^	4.90 ± 0.10^*b*^	6.70 ± 0.3^*b*^	0.78 ± 0.04^*a*^
GA_3_ 20	85 ± 2.6^*a*^	7.2 ± 0.38^*a*^	80 ± 2.30^*a*^	5.29 ± 0.12^*a*^	9.07 ± 0.3^*a*^	0.72 ± 0.03^*b*^
GA_3_ 50	99 ± 3.0^*a*^	7.5 ± 0.40^*a*^	81 ± 2.08^*a*^	5.17 ± 0.25^*a*^	11.5 ± 0.6^*a*^	0.71 ± 0.04^*b*^
GA_3_ 100	90 ± 2.8^*a*^	6.9 ± 0.26^*a*^	78 ± 1.15^*a*^	5.15 ± 0.20^*a*^	10.1 ± 0.5^*a*^	0.70 ± 0.03^*b*^
LSD (5%)	7.283	1.250	9.42	0.32	1.665	0.085

Control	30 ± 3.2^*b*^	6.5 ± 0.45^*b*^	69 ± 0.66^*b*^	4.90 ± 0.10^*c*^	6.70 ± 0.3^*c*^	0.78 ± 0.04^*a*^
NAA 5	74 ± 3.6^*a*^	7.8 ± 0.43^*a*^	79 ± 2.92^*a*^	4.95 ± 0.16^*b*^	9.76 ± 0.9^*b*^	0.73 ± 0.02^*b*^
NAA 10	80 ± 2.5^*a*^	8.0 ± 0.29^*a*^	82 ± 2.20^*a*^	5.12 ± 0.29^*a*^	10.7 ± 0.9^*a*^	0.72 ± 0.03^*b*^
NAA 20	76 ± 4.0^*a*^	7.5 ± 0.37^*a*^	80 ± 1.66^*a*^	5.09 ± 0.20^*b*^	9.70 ± 0.9^*b*^	0.71 ± 0.04^*b*^
LSD (5%)	5.47	1.43	9.27	0.35	0.836	0.0823

Control	30 ± 3.2^*b*^	6.5 ± 0.45^*b*^	69 ± 0.66^*b*^	4.90 ± 0.10^*b*^	6.70 ± 0.3^*b*^	0.78 ± 0.04^*b*^
2,4-D 5	79 ± 3.0^*a*^	6.9 ± 0.35^*a*^	78 ± 1.76^*a*^	4.99 ± 0.14^*a*^	8.70 ± 0.8^*b*^	0.73 ± 0.04^*b*^
2,4-D 10	83 ± 5.0^*a*^	7.0 ± 0.42^*a*^	75 ± 2.60^*a*^	5.15 ± 0.17^*a*^	8.90 ± 0.9^*b*^	0.74 ± 0.02^*b*^
2,4-D 20	72 ± 3.0^*a*^	6.7 ± 0.31^*a*^	74 ± 1.54^*a*^	4.85 ± 0.12^*b*^	7.26 ± 0.7^*b*^	0.74 ± 0.03^*b*^
LSD (5%)	5.57	1.33	9.53	0.38	1.582	0.093

Means (±SE) within the same column followed by the same letter do not differ significantly according to the LSD test at *α*′ = 0.05.

**Table 2:** Effects of growth regulators on TSS/acidity ratio, soluble carbohydrates, and total sugar content of wax apple fruits.

Treatment (mg/L)	TSS/acidity ratio	Glucose (%)	Fructose (%)	Inverted sugar (%)	Total sugar (mg/100 g)
Control	8.58 ± 1.3^*b*^	5.60 ± 0.29^*b*^	5.73 ± 0.14^*c*^	6.25 ± 0.7^*c*^	3.65 ± 0.47^*b*^
GA_3_ 20	12.6 ± 1.5^*a*^	7.00 ± 0.64^*a*^	7.08 ± 0.17^*b*^	7.37 ± 0.4^*b*^	5.57 ± 0.25^*a*^
GA_3_ 50	16.1 ± 1.7^*a*^	8.00 ± 0.20^*a*^	8.37 ± 0.15^*a*^	8.12 ± 0.4^*a*^	6.56 ± 0.23^*a*^
GA_3_ 100	14.4 ± 1.5^*a*^	7.60 ± 0.26^*a*^	8.18 ± 0.25^*a*^	7.93 ± 0.5^*a*^	5.82 ± 0.32^*a*^
LSD (5%)	2.548	1.065	1.081	1.319	0.526

Control	8.58 ± 1.3^*b*^	5.60 ± 0.29^*c*^	5.73 ± 0.14^*b*^	6.25 ± 0.70^*c*^	3.65 ± 0.47^*b*^
NAA 5	12.8 ± 2.0^*a*^	8.00 ± 0.23^*a*^	8.02 ± 0.15^*a*^	8.26 ± 0.60^*a*^	5.84 ± 0.20^*a*^
NAA 10	14.7 ± 2.1^*a*^	7.20 ± 0.32^*b*^	7.62 ± 0.10^*a*^	6.96 ± 0.43^*b*^	6.35 ± 0.17^*a*^
NAA 20	13.6 ± 1.7^*a*^	6.70 ± 0.18^*b*^	7.10 ± 0.27^*a*^	6.90 ± 0.45^*b*^	6.09 ± 0.23^*a*^
LSD (5%)	2.473	0.767	0.990	1.072	0.581

Control	8.58 ± 1.3^*b*^	5.60 ± 0.29^*a*^	5.73 ± 0.14^*b*^	6.25 ± 0.70^*a*^	3.65 ± 0.47^*b*^
2,4-D 5	12.8 ± 1.8^*a*^	6.25 ± 0.30^*a*^	6.30 ± 0.25^*a*^	6.50 ± 0.45^*a*^	5.83 ± 0.30^*a*^
2,4-D 10	13.7 ± 1.9^*a*^	6.16 ± 0.29^*a*^	6.26 ± 0.30^*a*^	6.40 ± 0.65^*a*^	6.20 ± 0.32^*a*^
2,4-D 20	10.1 ± 2.0^*a*^	6.00 ± 0.34^*a*^	5.80 ± 0.19^*a*^	6.17 ± 0.53^*a*^	4.81 ± 0.27^*b*^
LSD (5%)	2.872	0.653	0.782	0.890	0.672

Means (±SE) within the same column followed by the same letter do not differ significantly according to the LSD test at *α*′ = 0.05.

RETRACTED

**Table 3:** Effect of growth regulators on phytochemical properties and pigmentation of wax apple fruits.

Treatment (mg/L)	Ascorbic acid (mg/100 g)	Phenol mg GAE/100 g	Flavonoids (mg CE/100 g)	Chlorophyll (mg/L)	Anthocyanin (mg/100 g)	Carotenoid (*μ*g/g)
Control	5.1 ± 0.07^c^	311 ± 21.6^*c*^	18.5 ± 0.5^*b*^	0.63 ± 0.06^*a*^	24.3 ± 2.07^*c*^	5.97 ± 0.24^*b*^
GA_3_ 20	5.9 ± 0.06^*b*^	589 ± 51.4^*a*^	40.0 ± 2.0^*a*^	0.44 ± 0.02^*b*^	40.2 ± 3.13^b^	10.5 ± 0.36^*a*^
GA_3_ 50	6.6 ± 0.18^*a*^	535 ± 32.4^*b*^	45.0 ± 1.2^*a*^	0.24 ± 0.04^c^	46.0 ± 3.70^*a*^	11.3 ± 0.20^*a*^
GA_3_ 100	5.8 ± 0.19^*b*^	552 ± 99.5^*b*^	37.9 ± 1.7^*a*^	0.26 ± 0.02^*b*^	36.0 ± 2.83^*b*^	10.3 ± 0.12^*a*^
LSD (5%)	1.469	40.92	2.545	0.093	3.18	0.648

Control	5.1 ± 0.07^*c*^	311 ± 21.6^*c*^	18.5 ± 0.5^*b*^	0.63 ± 0.06^*a*^	24.3 ± 2.07^*c*^	5.97 ± 0. 24^*b*^
NAA 5	6.0 ± 0.10^*a*^	581 ± 25.3^*a*^	27.40 ± 1.8^*a*^	0.36 ± 0.03^*c*^	40.2 ± 0.25^*a*^	9.83 ± 0.40^*a*^
NAA 10	5.8 ± 0.14^*a*^	537 ± 40.7^*a*^	28.87 ± 1.8^*a*^	0.46 ± 0.05^*b*^	39.0 ± 1.34^*a*^	10.5 ± 0.32^*a*^
NAA 20	5.5 ± 0.16^*b*^	423 ± 55.6^*b*^	27.38 ± 1.2^*a*^	0.48 ± 0.04^*b*^	35.3 ± 1.46^*b*^	8.90 ± 0.25^*a*^
LSD (5%)	1.49	37.31	2.53	0.0987	5.440	0.625

Control	5.1 ± 0.07^*c*^	311 ± 21.6^*c*^	18.5 ± 0.5^*b*^	0.63 ± 0.06^*a*^	24.3 ± 2.07^*c*^	5.97 ± 0. 24^*b*^
2,4-D 5	5.6 ± 0.12^*a*^	525 ± 4.83^*a*^	27.31 ± 2.1^*a*^	0.44 ± 0.03^*b*^	36.0 ± 0.23^*b*^	9.00 ± 0.39^*a*^
2,4-D 10	5.4 ± 0.16^*a*^	415 ± 2.94^*b*^	25.57 ± 2.5^*a*^	0.48 ± 0.05^*b*^	35.0 ± 0.17^*a*^	7.80 ± 0.28^*a*^
2,4-D 20	5.1 ± 0.13^*b*^	303 ± 3.92^*c*^	22.83 ± 1.6^*a*^	0.45 ± 0.03^*b*^	28.0 ± 0.11^b^	7.50 ± 0.35^*a*^
LSD (5%)	1.52	41.54	3.934	5.47	5.574	0.643

Means (±SE) within the same column followed by the same letter do not differ significantly according to the LSD test at *α*′ = 0.05.
